The article "AGTH-Net: Attention-Based Graph Convolution-Guided Third-Order Hourglass Network for Sports Video Classification" was retracted in 2023. Reasons: unreliable results or conclusions; concerns about the data; concerns about the peer review; concerns about the citations.

# AGTH-Net: Attention-Based Graph Convolution-Guided Third-Order Hourglass Network for Sports Video Classification

**DOI:** 10.1155/2021/8517161

**Published:** 2021-07-06

**Authors:** Ming Gao, Weiwei Cai, Runmin Liu

**Affiliations:** ^1^College of Sports Science and Technology of Wuhan Sports University, Wuhan 430205, China; ^2^Central South University of Forestry and Technology, Changsha 410004, China; ^3^College of Sports Engineering and Information Technology, Wuhan Sports University, Wuhan 430079, China

## Abstract

As a hot research topic, sports video classification research has a wide range of applications in switched TV, video on demand, smart TV, and other fields and is closely related to people's lives. Under this background, sports video classification research has aroused great interest in people. However, the existing methods usually use manual video classification, which the workers themselves often influence. It is challenging to ensure the accuracy of the results, leading to the wrong classification. Due to these limitations, we introduce neural network technology to the automatic classification of sports. This paper proposed a novel attention-based graph convolution-guided third-order hourglass network (AGTH-Net) classification model. First, we designed a kind of figure convolution model based on the attention mechanism. The model is the key to introduce the attention mechanism for neighborhood node weights' allocation. It reduces the impact of error nodes in the neighborhood while avoiding manual weight assignment. Second, according to the sports complex video image characteristics, we use the third-order hourglass network structure. It is used for the extraction and fusion of multiscale characteristics of sports. In addition, in the hourglass, internal network residual-intensive modules are introduced, realizing characteristics in different levels of network transfer and reuse. It is helpful for maximum details to feature extracting and enhancing the network expression ability. Comparison and ablation experiments are also carried out to prove the effectiveness and superiority of the proposed algorithm.

## 1. Introduction

Sports video [1] is an essential resource in the video sports programs [2], which have hundreds of millions of loyal viewers in the world. Therefore, the classification of sports video research [3, 4] has become the focus of many researchers. The sports video classification technology can automatically classify the massive sports video data. Thus, it reduces people's workload and provides people with better spiritual enjoyment in daily life. It is also the basis of the automatic classification of intelligent broadcast and television. Therefore, the sports video classification technology can be widely used in sports video management [5], information retrieval [6], and query and offer a broad development prospect and great value.

The article "AGTH-Net: Attention-Based Graph Convolution-Guided Third-Order Hourglass Network for Sports Video Classification" was retracted in 2023. Reasons: unreliable results or conclusions; concerns about the data; concerns about the peer review; concerns about the citations.

Compared with other information resources, sports video resources are more popular with graphic, colorful, vivid, and engaging. However, video information contains a large amount of information, its structure is complex, and the number of videos grows exponentially every day. All these problems add many difficulties to the management and analysis of video data, and different users have different preferences for different types of videos. It is a difficult task to select the kind of video you need from the vast database. In real life, manual annotation can help users find the video content they are interested in, which can help improve the speed and save time to a certain extent. Manual labeling is prone to errors, and it is difficult to guarantee the accuracy of the labeling results. Suppose there is a deviation or wrong labeling. In that case, it will only be misleading to users. Wasting the user's time and energy, the results will do more harm than good. Of vast video annotation [7], the workload is enormous. It is impractical to use manual labeling, so it is not advisable to use manual labeling. In addition, the video watermarking technology [8] can be applied in video classification, such as in the video production phase to watermark or labels, which can help the user distinguish between different videos. However, after adding watermarks or labels, its robustness will be limited. It is easy to damage by artificial operation or accident. The information noted that the possibility of loss is very large. In order to facilitate users to efficiently browse and quickly find the videos they are interested in, as well as organize and manage the videos effectively, it has become an urgent problem to study the automatic classification [9], abstract generation [10], and semantic labeling of the massive video information with different styles.

With the progress of information technology, the classification research of sports video has made great progress in recent decades, which can be divided into three levels: type classification, event classification, and object classification. Event classification mainly classifies various scenes in specific videos into semantic events, such as the classification of free-kick, corner kick, shooting, and other events in football videos. Object classification mainly classifies the related objects in sports videos. For example, the video shot is divided into close-ups of human faces, spectators, athletes, etc. In contrast, type classification is used to distinguish the types of sports items, such as basketball, football, ping pong ball, etc. However, the research in this paper mainly focuses on the classification of sports types, as shown in Figure 1.

The article "AGTH-Net: Attention-Based Graph Convolution-Guided Third-Order Hourglass Network for Sports Video Classification" was retracted in 2023. Reasons: unreliable results or conclusions; concerns about the data; concerns about the peer review; concerns about the citations.

In this paper, the automatic classification of sports videos is our research focus. First, we introduced the convolutional neural network. The process of the convolution model is shown in Figure 1, where the importance of the neighborhood node is essential. The weight is set to a fixed, not considering the influence of different nodes on the classification task. However, a few neighborhood node weights were set out to cause the classification error. This paper designs a graph convolution [11] model based on an attention mechanism to solve the above problems. This model's key is to introduce an attention mechanism to carry out weight allocation to neighborhood nodes, reduce the influence of wrong nodes in the neighborhood, and save the work of manual weight allocation. This method can improve classification accuracy. Secondly, we also proposed the third-order hourglass network. We introduced the residual-density module inside it so that the features could be transmitted and reused at different levels of the network. As a result, the detailed features could be extracted to the maximum extent, and the expression ability of the network could be enhanced. Finally, the effectiveness and superiority of the proposed algorithm are proved by experiments.

The main contributions of this paper are as follows:

1. This paper proposes a novel three-order hourglass network classification model guided by the attention graph Convolution, which can automatically classify sports video images.
2. In this paper, a graph convolution model based on an attention mechanism is designed. This model's key is introducing an attention mechanism to carry out weight allocation to neighborhood nodes, reduce the influence of wrong nodes in the neighborhood, and avoid manual weight allocation.
3. We adopt the three-order hourglass network structure to extract and integrate multiscale sports features. In addition, the residual-density module is introduced inside the hourglass network to realize transmission and reuse of features in different levels of networks. It also extracts detailed features to the maximum extent and enhances the network expression ability.
4. We construct the sports image dataset and carry out the comparison and ablation experiments. The experimental results prove the effectiveness and superiority of the proposed algorithm.

The rest of the paper is organized according to the following pattern. First, in Section 2, related work is studied, followed by methodology in Section 3. Then, in Section 4, results and discussion are given in detail. Finally, Section 5 concludes the paper.

The article "AGTH-Net: Attention-Based Graph Convolution-Guided Third-Order Hourglass Network for Sports Video Classification" was retracted in 2023. Reasons: unreliable results or conclusions; concerns about the data; concerns about the peer review; concerns about the citations.

## 2. Related Work

With the advancement of information technology, the classification research of sports videos has made considerable progress in recent decades. Some scholars have proposed many methods and models in the field of video classification. Babaguchi et al. [12] used principal components to reduce the dimension of video visual and audio features to describe the video content and then used the time series of motion features to distinguish the classification of action events in football video. According to the field area and field distribution characteristics, the football video shot classification, event detection, and video summaries are realized. Ma et al. [13] realized the classification of simple sports in sports videos by detecting some motion patterns in video frames, such as running, jumping, serving shots, panning, and zooming. Liu et al. [14] realized the classification of videos by separating the target objects and other information in the video. When the video background is relatively single, and there are few occlusion areas between objects, the effect is good. However, when the video background is complex or the target, the experimental results are not accurate enough when there is much overlap. Truong et al. [15] extracted video editing, color, and motion features from the literature. They realized the classification of sports and other kinds of videos by constructing the idea of a decision tree. However, due to the restriction of a decision tree, the experimental results often converge to the optimal local solution rather than the whole optimal solution, resulting in specific errors. Xavier et al. [16] extracted the feature vectors composed of video motion and primary color information. They established a classifier based on HMM model to classify sports videos into various items. The experimental accuracy is high, but using HMM as a classifier requires a large number of training samples and observation sequences, which will lead to an increase in the amount of calculation. Geetha et al. [9] proposed a video classification method based on HMM and realized video classification by selecting relatively simple features. Moreover, the establishment of its classification model often relies on a large number of training data, which leads to a significant increase in the workload in the actual work. In addition, the observation sequence of HMM model also needs to be long enough, so the calculation amount will also increase.

In terms of the classification model based on machine learning, there are four kinds of balls. Watcharapinchai et al. [17] proposed a classification method based on a color autocorrelation graph to classify sports video visual types. The average accuracy of the SVM classifier was higher than the others. Through comparison, it was proved that the classification effect of SVM was better than that of the PCA neural network. Mohan et al. [18] proposed the feature of edge direction and edge intensity. They designed a classifier based on a self-associated neural network to classify sports videos. Based on the combination of SVM and neural networks [19–23], the classification accuracy is high. However, the algorithm complexity of the joint classifier is high. The fusion algorithm of the two features is complex, and the computation is also significant. Capodiferro et al. [24] used SVM to classify Olympic sports videos into different sports events by integrating multiple features of color, brightness, and texture of video frames. Since the experimental materials are aged sports video sets, the generalization ability needs to be enhanced. In addition, some scholars have also begun to introduce deep learning techniques [25–29] to sports classification tasks.

The article "AGTH-Net: Attention-Based Graph Convolution-Guided Third-Order Hourglass Network for Sports Video Classification" was retracted in 2023. Reasons: unreliable results or conclusions; concerns about the data; concerns about the peer review; concerns about the citations.

## 3. Methodology

In this section, the following subsections attention-based graph convolution, third-order hourglass networks, and residual dense module are discussed in detail.

Figure 2 is the overall architecture of our sports classification model. This paper designs a graph convolution model based on the attention mechanism. The key of the model is to introduce the attention mechanism to assign weights to neighboring nodes, reduce the influence of wrong nodes in the neighborhood, and avoid manually assigning weights. Secondly, we adopt a three-level hourglass network structure to extract and fuse multiscale sports features because of sports video images' complex and diverse characteristics. In addition, inside the hourglass network, a residual-intensive module is introduced to extract features in different levels of networks. It realizes transmission and reuses, extracts detailed features to the maximum extent, and enhances network expression ability. Next, the AGTH-Net algorithm will be explained in detail.

### 3.1. Attention-Based Graph Convolution

In recent years, the classification model is based on an attention mechanism that has developed vigorously. It allows the model to focus on the critical part of the feature space and distinguish irrelevant information. It can also increase the sensitivity to features that contain more useful information. Considering the complex and changeable background environment of sports image data, we add the attention mechanism to the graph convolution to effectively filter out the influence of harmful information. Thereby, it is helping to extract the deep semantic features of sports images using the proposed model. As shown in Figure 3, the attention mechanism can reduce the impact of unfavorable information.

The article "AGTH-Net: Attention-Based Graph Convolution-Guided Third-Order Hourglass Network for Sports Video Classification" was retracted in 2023. Reasons: unreliable results or conclusions; concerns about the data; concerns about the peer review; concerns about the citations.

The graph convolution model can act on each node and extract the sports video image's in-depth features by continuously collecting each neighborhood node's information. Compared with the convolutional neural network, the convolutional graph network can deal with irregular graph data, which can overcome the defects of the fixed convolution kernel. Because of the complex and changeable background of sports video images, we need to identify potentially harmful information of neighboring nodes. It effectively extracts the relevant information from them and reduces the impact of harmful information. We introduce the attention mechanism into the graph convolution model. It can explain how the neighborhood nodes in the airspace affect the central node classification task. Thereby, it improves the interpretability of the graph convolution model and provides an interpretable basis for the model in the classification of sports video images.

The attention mechanism used in this paper is the self-attention mechanism (as shown in Figure 4). The input of the layer is a set of node features *H*={*h*_1_, *h*_2_,…, *h*_*i*_},  *h*_*i*_ ∈ *R*^*F*^, where *N* is the number of nodes and *F* is the dimension of each node feature. This layer will generate a set of new node features *H*′={*h*_1_′, *h*_2_′,…, *h*_*i*_′},  *h*_*i*_′ ∈ *R*^*F*′^ as its output. In order to transform the input features into higher-level features to obtain sufficient expressive ability, the model needs at least one learnable linear transformation. Therefore, in the first step, we apply the linear transformation parameterized by the weight matrix *W* ∈ *R*^*F*×*F*′^ to each node and then execute the self-attention mechanism *a* : *R*^*F*^ × *R*^*F*′^⟶*R* on each node to calculate the attention coefficient:

(1) $$\begin{array}{c} e_{ij}=a\left(W{\overset{⟶}{h}}_{i},W{\overset{⟶}{h}}_{i}^{\prime }\right), \end{array}$$

where *e*_*ij*_ represents the importance of the characteristics of the node *j* to node *i*. In the general attention model, the model allows each node to participate in the attention calculation of any other node, which will cause a lot of computational overhead and discarding all structural information. We incorporate the graph structure into the mechanism by performing mask attention. This chapter only calculates *e*_*ij*_(*j* ∈ *N*_*i*_) of the node, where *N*_*i*_ is the neighborhood of the node *i* in the graph. In all the experiments in this article, these *j* nodes will happen to be the first-order neighbors of node *i*. In order to make the coefficients easy to compare on different nodes in the whole range, we use the softmax function to normalize all the selected *j*:

(2) $$\begin{array}{c} a_{ij}=\text{softmax}\left(e_{ij}\right)\\ =\frac{\text{exp}\left(e_{ij}\right)}{\sum_{k\in N_{i}}e_{ik}}. \end{array}$$

The full expansion of the coefficient calculated by the attention mechanism can be expressed as

(3) aij=expReLUa⟶TWh⟶i∘Wh⟶i′∑k∈NiexpReLUa⟶TWh⟶i∘Wh⟶i′,

where *T* stands for transpose and ∘ stands for connection operation. When the normalized attention coefficient is obtained, it can be used to calculate the features corresponding to them as the final output feature of each node:

(4) $$\begin{array}{c} {\overset{⟶}{h}}_{i}^{\prime }=\sigma \left(\sum_{j\in N_{i}}a_{ij}W{\overset{⟶}{h}}_{j}\right). \end{array}$$

The article "AGTH-Net: Attention-Based Graph Convolution-Guided Third-Order Hourglass Network for Sports Video Classification" was retracted in 2023. Reasons: unreliable results or conclusions; concerns about the data; concerns about the peer review; concerns about the citations.

### 3.2. Third-Order Hourglass Networks

This section will specifically introduce the third-order hourglass network structure and residual-intensive module proposed in this paper. The hourglass structure is an approximately symmetrical structure, which can be defined as the following equation:

(5) $$\begin{array}{c} {\text{Hourglass}}_{i}=F_{u}^{i}\left(F_{d}^{i}\left(X;\theta_{d}\right);\theta_{u}\right)+\sum_{j=1}^{i}F_{d}^{j-1}\left(X;\theta_{d}\right), \end{array}$$

where *X* is the input data, *F*_*d*_(*X*; *θ*_*d*_) is the process of subsampling the input data, *F*_*u*_(*X*; *θ*_*u*_) is the process of sampling up data, and *i*, *j* represent the number of layers of up- and downsampling. The hourglass structure output is the fusion of the features obtained by up- and downsampling processing and the features obtained by the residual network. The lower sampling layer can improve the focus area of the network and obtain higher dimensional information, which is conducive to the network better to distinguish the information of different depths and scales. Upsampling amplifies the image features through deconvolution, forming a cross-layer structure, which can better retain the details and edge information of the image. The number of upper and lower sampling layers can be adjusted according to the needs of data processing. The introduction of the residual network can integrate local details and high-dimensional depth information, which is favorable to obtaining deep semantic information of sports images in a complex environment.

The third-order hourglass network can effectively extract low-dimensional and high-dimensional information at different scales. Low-dimensional information ensures the accuracy of feature information, and high-dimensional information can better process global and depth information. In order to make better use of multiscale feature information, we use attention-based graph convolution to fuse features of different scales to improve the utilization of multiscale features, as shown in Figure 5.

The article "AGTH-Net: Attention-Based Graph Convolution-Guided Third-Order Hourglass Network for Sports Video Classification" was retracted in 2023. Reasons: unreliable results or conclusions; concerns about the data; concerns about the peer review; concerns about the citations.

### 3.3. Residual Dense Module

In order to better perform deep feature extraction on sports images and improve the classification accuracy, we introduced a residual-intensive module (as shown in Figure 6).

The residual dense module is composed of a residual network and a densely connected network. The residual network can effectively help the characteristic information to be transmitted to deeper network information. From the perspective of the characteristic layer, the dense network connects any two layers of the network to maximize. The network's information connection enables each layer of the network to receive the feature input from all the previous layers, which can effectively suppress gradient dissipation in the training process. Because the dense network realizes feature reuse and transfer, fewer features are also fully utilized. The model size is also smaller. By combining the characteristics of the above two networks, the dense residual network can be defined as

(6) $$\begin{array}{c} x_{l+1}=x_{l}+F\left(G_{d}\left(\left[x_{0},x_{1},\ldots ,x_{d}\right]\right),\left[W_{0},W_{1},\ldots ,W_{d}\right]\right), \end{array}$$

where *x*_*l*_ and *x*_*l*+1_ are the *l*-th and *l*+1 layers of the dense residual network and [*x*_0_, *x*_1_,…, *x*_*d*_] and [*W*_0_, *W*_1_,…, *W*_*d*_] are the sum of the parameters corresponding to all convolutional layers in the residual dense network Characteristic information. *F* is the residual network feature extraction process and *G* is the dense network.

## 4. Experiments and Results

This section discusses experimental setup, datasets, evaluation methods, and experimental results discussed in detail.

### 4.1. Experimental Setup

To evaluate the AGTH-Net algorithm in this paper fairly, all experiments in this paper are carried out in the same environment. The entire network runs under the Keas framework, Windows system 10, and the graphics card is NVIDIA GTX1080 GPU (8 GB). The training image dataset has an image size of 224 × 224 pixels as input, using *a*  *da*  *m* optimization, the initial learning rate is 1 × 10^−3^, and the batch size is 32. There are 300 epochs in the training process, and the learning rate is reduced by half every 10 epochs.

### 4.2. Datasets

In the study of sports classification, there is no unified video database to verify the performance of each classification algorithm. Therefore, a standard test database will have a crucial impact on the experimental results. In the experiment, we used Python to write a crawler program. We crawled a total of 2200 sports images from the Internet, including 799 football images, 689 swimming images, and 712 table tennis images, as shown in Figure 7 and Table 1.

The article "AGTH-Net: Attention-Based Graph Convolution-Guided Third-Order Hourglass Network for Sports Video Classification" was retracted in 2023. Reasons: unreliable results or conclusions; concerns about the data; concerns about the peer review; concerns about the citations.

Before input to the neural network for training, all images are preprocessed into a size of 224 × 224. Then, we divide 75% of them into the training set, with a total of 1650 images, and the remaining 25% as the test set, with a total of 550 images.

### 4.3. Evaluation Methods

Since the research in this article is mainly classification and recognition, we use precision, recall, and *F*_1_-score to evaluate the AGTH-Net algorithm. The calculation equations of the three evaluation indicators are as follows:

(7) $$\begin{array}{c} \text{precision}=\frac{\text{TP}}{\text{TP}+\text{FP}},\\ \text{recall}=\frac{\text{TP}}{\text{TP}+\text{FN}},\\ F_{1}=\frac{2\times \text{precision}\times \text{recall}}{\text{precision}+\text{recall}}, \end{array}$$

where TP means the sample is positive and predicted to be positive, TN means the sample is negative and predicted to be negative, FP means the sample is negative but predicted to be positive, and FN means the sample is positive but predicted to be negative.

### 4.4. Experimental Results

#### 4.4.1. Classification Performance

It can be seen from Table 2 and Figure 8 that, in the classification of various types of sports, the precision of football, swimming, and table tennis reaches or exceeds 93%. On the other hand, the precision of table tennis is relatively low, and both swimming and football reach or exceed 95%. Thus, the data shows that the AGTH-Net algorithm established in this paper is effective for sports video classification.

Although the classification of recall in football and table tennis is only about 92%, further subjective observation on video clips shows that many misjudgment clips are shot clips composed of close-ups of spectators, coaches, referees, or athletes. For such footage, people's subjective judgment will also misjudge. Therefore, the category judgment of such shots should be further improved with the help of the domain knowledge model. However, suppose this type of video clip is removed. In that case, the AGTH-NET algorithm proposed in this paper will be improved to a certain extent. In addition, we also give a confusion matrix for classification performance, as shown in Figure 9.

#### 4.4.2. Comparative Experiment

To verify the superiority of the AGTH-Net algorithm, we conducted comparative experiments with the four well-known methods of SVM, BP network, GoogleNet, and AlexNet. The experimental results are shown in Table 3.

The article "AGTH-Net: Attention-Based Graph Convolution-Guided Third-Order Hourglass Network for Sports Video Classification" was retracted in 2023. Reasons: unreliable results or conclusions; concerns about the data; concerns about the peer review; concerns about the citations.

It can be seen from Table 3 and Figure 10 that the AGTH-Net algorithm has achieved the best performance. It is 5.1%–26.8% higher than the other four methods in football recognition, 4.2%–30.5% higher than the other four methods in swimming, and 4.3%–33.3% higher than the other four methods on table tennis. It fully proves the superiority of the AGTH-Net algorithm.

#### 4.4.3. Ablation Experiment

To verify the influence of the attention-based graph convolution, we have used the third-order hourglass network and the residual dense module on the classification performance. An ablation experiment is carried out in this section. AGC means that only attention-based graph convolution is used. TOH means that only third-order hourglass networks are used. In contrast, TOH-RD means that both third-order hourglass networks and residual-intensive modules are used. The attention-based graph convolution is not used. The experimental results are shown in Table 4.

It can be seen from Table 4 and Figure 11 that a single AGC is better than TOH. It proves that graph convolution can effectively provide deep semantic information in a complex background environment, and TOH-RD is better than AGC and TOH. Furthermore, it proves that the residual error is third-order. The hourglass network can extract dimensional and high-dimensional information of different scales. Low-dimensional information ensures the accuracy of feature information, and high-dimensional information can better process global and depth information. At the same time, we found that even a single module is better than the compared group method, which once again proves the effectiveness and superiority of the AGTH-Net algorithm.

## 5. Conclusion

In this paper, we introduce neural network technology to the automatic classification of sports. This paper proposes novel attention to convolution-guided third-order hourglass network classification model. First of all, this paper designed a kind of figure convolution model based on the attention mechanism. The model is the key to introducing an attention mechanism for neighborhood node weights allocation and reducing the effect of the error node neighborhood. At the same time, manual weight allocation is avoided. Second, according to the sports complex video image characteristics, we use the third-order hourglass network structure to extract and fuse multiscale sports characteristics. In addition, the hourglass internal network introduces residual-intensive modules and realization characteristics in the different level network transfer and reuse. Therefore, it maximizes details feature extracting and enhances the network expression ability. Finally, we conducted a performance test experiment, and the comparison and ablation experiment results proved the effectiveness and superiority of the AGTH-NET algorithm.

The article "AGTH-Net: Attention-Based Graph Convolution-Guided Third-Order Hourglass Network for Sports Video Classification" was retracted in 2023. Reasons: unreliable results or conclusions; concerns about the data; concerns about the peer review; concerns about the citations.

## Figures and Tables

**Figure 1:** Examples of sports video classification.

**Figure 2:** The overall architecture of the AGTH-Net algorithm.

**Figure 3:** Schematic diagram of the attention mechanism screening feature information: (a) no attention; (b) attention.

**Figure 4:** Schematic diagram of the self-attention mechanism.

**Figure 5:** The attention-based third-order hourglass network framework; AGC represents the attention-based graph convolution.

**Figure 6:** Schematic diagram of the residual dense module.

**Figure 7:** Examples of datasets.

**Figure 8:** Classification results of sports videos. (a) Classification and recognition results of football videos. (b) Classification and recognition results of swimming videos.

**Figure 9:** Confusion matrix.

**Figure 10:** Histogram of comparison results of different methods.

**Figure 11:** Visualization of the results of the ablation experiment. (a) Football (precision). (b) Swimming (precision). (c) Table tennis (precision).

**Table 1:** Dataset.

Sports category	Source	Number
Football	Internet	799
Swimming	Internet	689
Table tennis	Internet	712

**Table 2:** Classification performance of the AGTH-Net algorithm.

Sports category	Precision	Recall	*F*_1_-score
Football	0.97	0.92	0.96
Swimming	0.95	0.96	0.95
Table tennis	0.93	0.92	0.96

**Table 3:** Comparison results of different methods (precision).

Sports category	Football	Swimming	Table tennis
SVM	0.71	0.66	0.62
BP	0.79	0.75	0.72
GoogleNet	0.91	0.91	0.89
AlexNet	0.92	0.91	0.89
AGTH-Net	0.97	0.95	0.93

**Table 4:** Results of ablation experiments.

Sports category	Football	Swimming	Table tennis
AGC	0.92	0.90	0.92
TOH	0.91	0.89	0.91
TOH-RD	0.93	0.92	0.92
AGTH-Net	0.97	0.95	0.93

## Data Availability

The data used to support the findings of this study are available from the corresponding author upon request.
